The article "Impact of cardiovascular and metabolic diseases on the severity of COVID-19: a systematic review and meta-analysis" was published in 2020. Journal: Aging (Albany NY).

# Impact of cardiovascular and metabolic diseases on the severity of COVID-19: a systematic review and meta-analysis

**DOI:** 10.18632/aging.103991

**Published:** 2020-11-16

**Authors:** Meng Meng, Qianwen Zhao, Rahul Kumar, Chen Bai, Yunlei Deng, Bo Wan

**Affiliations:** 1 Digestion Center, Beijing Hospital of Traditional Chinese Medicine, Capital Medical University, Beijing, China; 2 Department of Gastroenterology and Hepatology, Sichuan University-Oxford University Huaxi Gastrointestinal Cancer Centre, West China Hospital, Sichuan University, Chengdu, China; 3 Department of Gastroenterology and Hepatology, Changi General Hospital, Singapore; 4 Beijing University of Chinese Medicine, Beijing, China; 5 Department of Nephrology, The Third People’s Hospital of Chengdu, Chengdu, China; 6 Centre for Stem Cells and Regenerative Medicine, King’s College London, Guy’s Hospital, Great Maze Pond, London, UK

**Keywords:** COVID-19, 2019-nCoV, coronary heart disease, hypertension, diabetes, severe pneumonia

## Abstract

We examined the effects of coronary heart disease (CHD), hypertension and diabetes on the development of severe COVID-19. We performed a comprehensive, systematic literature search for studies published between December 2019 and July 5, 2020 in five databases. The prevalence of severe COVID-19 in patients with CHD, hypertension and diabetes was evaluated through a meta-analysis. Thirty-five articles with 8,170 patients were included, and all the available studies were case series. The pooled odds ratio for the development of severe COVID-19 was 3.21 for patients with CHD (fixed-effects model, 95% CI: 2.58-3.99), 2.27 for patients with hypertension (random-effects model, 95% CI: 1.79-2.90) and 2.34 for patients with diabetes (random-effects model, 95% CI: 1.79-3.05). The heterogeneity of the studies was moderate for the effect of CHD on COVID-19 severity, but was high for the effects of diabetes and hypertension. Funnel plots and Egger’s tests revealed no publication bias in the CHD and hypertension analyses, but suggested publication bias in the diabetes analysis. This bias was corrected using the trim-and-fill method, and was ultimately found to have no effect on the results. Our findings suggest patients with CHD, hypertension and diabetes are at greater risk for developing severe COVID-19 than those without these conditions.

## INTRODUCTION

Coronavirus disease 2019 (COVID-19) is a potentially severe acute respiratory infection caused by severe acute respiratory syndrome coronavirus 2 (SARS-CoV-2), which was newly discovered in December 2019 [1]. By March 2020, the outbreak had spread to more than 200 countries, rapidly evolving into a pandemic. At the time of the World Health Organization’s situation report on July 12, 2020, over 12 million laboratory-confirmed cases and 550,000 deaths had been documented globally.

The article "Impact of cardiovascular and metabolic diseases on the severity of COVID-19: a systematic review and meta-analysis" was published in 2020. Journal: Aging (Albany NY).

Elderly patients and those with pre-existing health conditions are more likely to progress to severe COVID-19 [2, 3]. Coronary heart disease (CHD), hypertension and diabetes are the most prevalent diseases worldwide, as their prevalence increases with advancing age. A previous meta-analysis indicated that patients with pre-existing cardiovascular and metabolic diseases may be at increased risk for intensive care unit admission and poor outcomes upon infection with SARS-CoV-2 [4]. However, the analysis only included six studies with relatively high heterogeneity, raising some questions about the reliability of the conclusions. Therefore, the risk of COVID-19 progression in patients with cardiovascular and metabolic diseases requires further investigation.

Herein, we conducted a meta-analysis to investigate the relationship between severe COVID-19 and underlying CHD, hypertension and diabetes.

## RESULTS

### Research study selection and quality assessment

Based on our search strategy, 29,617 studies were retrieved from five online databases. Duplicate records were deleted, such that 18,924 records were retained. Of these, 18,852 articles were excluded based on their titles and abstracts, and 37 of the remaining 72 articles were deleted for various other reasons (Figure 1). Ultimately, 35 articles (one in Chinese and the remainder in English) were included in the meta-analysis [5–39]. The characteristics and patient demographics of the included studies are shown in Table 1. The quality of the included articles was also evaluated, as shown in Table 2. The Methodological Index for Non-Randomized Studies (MINORS) scores of the studies ranged from 10-14.

**Figure 1:** **Flow diagram of the literature screening.**

**Table 1:** Characteristics and demographic data of the included studies.

**author**	**year**	**origin**	**language**	**outcome**	**mean age**	**male n(%)**	**severe cases/total cases —no./total no. (%)**	**severe cases in Coronary heart disease/total cases of Coronary heart disease —no./total no. (%)**	**severe cases in Hypertension /total cases of Hypertension —no./total no. (%)**	**severe cases in Diabetes/total cases of Diabetes —no./total no. (%)**
COVID-19 Australia Incident Room Surveillance Team	2020	Australia	English	ICU	58.67	306(51.00%)	157/600(26.17%)	NR	NR	38/107(35.51%)
D. Colombi	2020	Italy	English	ICU	68.00	177(75.00%)	108/236(45.76%)	77/127(60.63%)	NR	22/37(59.46%)
M. Choi	2020	South Korea	English	Composite End Point	33.33	214(73.04%)	36/293(12.29%)	NR	9/29(31.03%)	10/21(47.62%)
Y. Deng	2020	China	English	Death	55.83	124(55.11%)	109/225(48.44%)	13/17(76.47%)	40/58(68.97%)	17/26(65.83%)
X. Fang	2020	China	Chinese	Composite End Point	45.10	45(56.96%)	24/79(30.38%)	2/3(66.67%)	11/16(68.75%)	4/8(50.00%)
P. Goyal	2020	US	English	Composite End Point	61.50	238(60.60%)	130/393(33.08%)	NR	70/197(35.53%)	36/99(36.36%)
W. Guan	2020	China	English	Composite End Point	46.67	640(58.23%)	67/1099(6.10%)	10/27(37.04%)	41/165(24.85%)	18/81(22.22%)
Y. Gao	2020	China	English	Composite End Point	44.08	26(60.47%)	15/43(34.88%)	1/3(33.33%)	6/13(46.15%)	6/7(85.71%)
C. Huang	2020	China	English	ICU	49.33	30(73.17%)	13/41(31.71%)	3/6(50.00%)	2/6(33.33%)	1/8(12.50%)
S. Huang	2020	China	English	ICU	NR	NR	51/310(16.45%)	NR	27/113(23.89%)	NR
K. Li	2020	China	English	Composite End Point	45.50	44 (53.00%)	25/83(30.12%)	1/1(100.00%)	2/5(40.00%)	7/7(100.00%)
W. Liu	2020	China	English	Composite End Point	42.67	39 (50.00%)	11/78(14.10%)	NR	2/8(25.00%)	2/5(40.00%)
X. Li	2020	China	English	Composite End Point	59.00	279(50.90%)	269/548(49.09%)	28/34(82.35%)	104/166(62.65%)	52/83(62.65%)
Y. Liu	2020	China	English	Composite End Point	53.67	8(66.67%)	3/12(25.00%)	¼(25.00%)	1/3(33.33%)	1/2(50.00%)
F. Montastruc	2020	France	English	Composite End Point	57.47	76(79.17%)	71/96(73.96%)	NR	32/43(74.42%)	16/27(59.26%)
L. Myers	2020	US	English	ICU	61.33	212(56.20%)	113/377(29.97%)	NR	58/164(35.37%)	45/118(38.14%)
B. Nowak	2020	Poland	English	Death	63.70	87 (51.50%)	46/169(27.22%)	22/58(37.93%)	27/80(33.75%)	16/32(50.00%)
Y. Nie	2020	China	English	Composite End Point	43.00	367(56.03%)	72/655(10.99%)	8/70(11.43%)	5/60(8.33%)	1/12(8.33%)
C. Qin	2020	China	English	Composite End Point	57.33	235(52.00%)	286/452(63.27%)	24/27(88.89%)	105/135(77.78%)	53/75(70.67%)
A. Simonnet	2020	France	English	Composite End Point	60.33	90(73.00%)	85/124(68.55%)	NR	48/60(80.00%)	23/28(82.14%)
C. Wu	2020	China	English	Composite End Point	51.33	128(63.68%)	84/201(41.79%)	5/8(62.50%)	23/39(58.97%)	16/22(72.73%)
D. Wang	2020	China	English	ICU	55.33	75(54.35%)	36/138(26.09%)	9/20(45.00%)	21/43(48.84%)	8/14(57.14%)
F. Wang	2020	China	English	ICU	68.60	21(75.00%)	14/28(50.00%)	4/4(100.00%)	10/15(66.67%)	NR
L. Wang	2020	China	English	Composite End Point	53.67	67(57.80%)	57/116(49.14%)	NR	20/43(46.51%)	10/18(55.56%)
S. Wan	2020	China	English	Composite End Point	46.00	72(53.30%)	40/135(29.63%)	6/7(85.71%)	4/13(30.77%)	9/12(75.00%)
X. Wang	2020	China	English	Composite End Point	49.00	59(45.04%)	69/131(52.67%)	2/3(66.67%)	¾(75.00%)	2/2(100.00%)
Y. Wang	2020	China	English	Death	62.67	165(47.97%)	133/344(38.66%)	22/40(55.00%)	69/141(48.94%)	30/64(46.88%)
Z. Wang	2020	China	English	Composite End Point	46.33	32(46.38%)	14/69(20.29%)	5/8(62.50%)	5/9(55.56%)	6/7(85.71%)
Y. Xie	2020	China	English	Composite End Point	64.00	27(43.55%)	24/62(38.71%)	17/33(51.52%)	NR	NR
Z. Xiong	2020	China	English	Composite End Point	50.67	214(50.83%)	59/421(14.01%)	NR	8/44(18.18%)	3/13(23.08%)
L. Yang	2020	China	English	ICU	55.00	98(49.00%)	29/200(14.50%)	1/11(9.09%)	9/45(20.00%)	4/21(19.05%)
X. Yang	2020	China	English	Death	59.70	35(67.31%)	32/52(61.54%)	3/5(60.00%)	NR	7/9(77.78%)
F. Zhou	2020	China	English	Death	56.33	119(62.30%)	54/191(28.27%)	13/15(86.67%)	26/58(44.83%)	17/36(47.22%)
J. Zhang	2020	China	English	Composite End Point	56.33	71(50.71%)	58/140(41.43%)	4/7(57.14%)	22/42(52.38%)	8/17(47.06%)
J. Zhao	2020	China	English	Composite End Point	51.00	14(48.28%)	21/29(72.41%)	9/10(90.00%)	NR	7/7(100.00%)

* Composite end point in original studies was defined as SpO2<90% or requirement of an intensive care or the use of mechanical ventilation, or death.

The article "Impact of cardiovascular and metabolic diseases on the severity of COVID-19: a systematic review and meta-analysis" was published in 2020. Journal: Aging (Albany NY).

**Table 2:** Bias risk assessment.

**Study**	**1**	**2**	**3**	**4**	**5**	**6**	**7**	**8**	**Score**
COVID-19 Australia Incident Room Surveillance Team	2	2	2	2	2	1	2	0	13
D. Colombi	2	2	2	2	2	0	0	0	10
M. Choi	2	2	2	2	2	2	1	0	13
Y. Deng	2	2	2	2	2	0	0	0	10
X. Fang	2	2	2	2	2	1	2	0	13
P. Goyal	2	2	2	2	2	0	0	0	10
W. Guan	2	2	2	2	2	0	0	0	10
Y. Gao	2	2	2	2	2	0	0	0	10
C. Huang	2	2	2	2	2	1	2	0	13
S. Huang	2	2	2	2	2	0	0	0	10
K. Li	2	2	2	2	2	0	0	0	10
W. Liu	2	2	2	2	2	1	2	0	13
X. Li	2	2	2	2	2	2	1	0	13
Y. Liu	2	2	2	2	2	0	0	0	10
F. Montastruc	2	2	2	2	2	0	0	0	10
L. Myers	2	2	2	2	2	2	2	0	14
B. Nowak	2	2	2	2	2	0	0	0	10
Y. Nie	2	2	2	2	2	2	1	0	13
C. Qin	2	2	2	2	2	0	0	0	10
A. Simonnet	2	2	2	2	2	0	0	0	10
C. Wu	2	2	2	2	2	0	0	0	10
D. Wang	2	2	2	2	2	1	2	0	13
F. Wang	2	2	2	2	2	2	1	0	13
L. Wang	2	2	2	2	2	0	0	0	10
S. Wan	2	2	2	2	2	0	0	0	10
X. Wang	2	2	2	2	2	0	0	0	10
Y. Wang	2	2	2	2	2	0	0	0	10
Z. Wang	2	2	2	2	2	1	2	0	13
Y. Xie	2	2	2	2	2	0	0	0	10
Z. Xiong	2	2	2	2	2	0	0	0	10
L. Yang	2	2	2	2	2	0	0	0	10
X. Yang	2	2	2	2	2	1	2	0	13
F. Zhou	2	2	2	2	2	0	0	0	10
J. Zhang	2	2	2	2	2	0	0	0	10
J. Zhao	2	2	2	2	2	2	2	0	14

1 A clearly stated aim;

2 Inclusion of consecutive patients;

3 Prospective collection of data;

4 Endpoints appropriate to the aim of the study;

5 Unbiased assessment of the study endpoint;

6 Follow-up period appropriate to the aim of the study;

7 Loss to follow up less than 5%;

8 Prospective calculation of the study size.

The items are scored 0 (not reported), 1 (reported but inadequate) or 2 (reported and adequate). The global ideal score being 16 for non-comparative studies.

### Characteristics of the included studies

Of the 8,170 patients in the 35 studies included in this meta-analysis, 2,415 patients (29.56%) met the criteria for severe COVID-19. Ten studies did not report the prevalence of CHD [9, 18, 19, 22, 24, 27, 31, 32, 35, 37], five studies did not report the prevalence of hypertension [14, 20, 32, 36, 39] and three studies did not report the prevalence of diabetes [24, 34, 36]. The remaining studies reported the prevalence of CHD, hypertension and diabetes in their respective patient pools. In the original data, the prevalence of each disease in severe or non-severe COVID-19 patients was presented. To better visualize the risk, we converted the data and presented the incidence of severe COVID-19 in the populations with CHD, hypertension and diabetes.

The article "Impact of cardiovascular and metabolic diseases on the severity of COVID-19: a systematic review and meta-analysis" was published in 2020. Journal: Aging (Albany NY).

The patients in the studies were from China (27 studies), Italy (1 study), the United States (2 studies), France (2 studies), Australia (1 study), Poland (1 study) and South Korea (1 study). The average age of the patients ranged from 33.3 to 68.6 years. The incidences of CHD, hypertension and diabetes in all the included patients were 6.71%, 22.24% and 12.55%, respectively. The incidences of CHD, hypertension and diabetes in severe patients were 12.01%, 33.54% and 20.50%, respectively. Men were more likely than women to develop severe pneumonia (61.55% of severe cases were men).

### CHD and the severity of COVID-19

A forest plot was used to evaluate the association between CHD and COVID-19 severity. In the forest plot, the odds ratio (OR) indicates the strength of the association between the basic disease and the severity of COVID-19. The vertical line indicating no effect crosses the horizontal axis at an OR of 1. The length of each horizontal line represents the range of the 95% confidence interval (CI) of the corresponding study. The small square in the middle of the line demonstrates the position of the OR, and the size of the square represents the weight of the study. If the combined OR for all the studies does not intersect with the vertical line of no effect, the results are statistically significant.

Twenty-five studies reported the relationship between CHD and the severity of COVID-19. The pooled OR is displayed in Figure 2A, which demonstrates that CHD increased the risk of severe COVID-19 at least three-fold (fixed-effects model, OR=3.21, 95% CI: 2.58-3.99). The heterogeneity among the included studies was moderate (I^2^=38%, p=0.03).

**Figure 2:** (**A**) Forest plot for CHD. (**B**) Funnel plot for CHD.

A funnel plot and Egger’s test were used to evaluate publication bias. In a funnel plot, studies with large sample sizes and high precision are distributed at the top of the plot and concentrated toward the center, while studies with small sample sizes and relatively low accuracy are distributed in the middle and lower parts of the plot in a symmetrical arrangement. Egger’s test (p=0.7511) and the funnel plot indicated no publication bias for the studies examining the association between CHD and COVID-19 severity (Figure 2B).

The article "Impact of cardiovascular and metabolic diseases on the severity of COVID-19: a systematic review and meta-analysis" was published in 2020. Journal: Aging (Albany NY).

### Hypertension and the severity of COVID-19

Thirty studies reported the relationship between hypertension and the severity of COVID-19. The duration of hypertension was not reported in most studies. The pooled OR is depicted in Figure 3A, which demonstrates that hypertension increased the risk of severe COVID-19 at least two-fold (random-effects model, OR=2.27, 95% CI: 1.79-2.90). The heterogeneity among the studies was high (I^2^=65%, p<0.01). A sensitivity analysis revealed that the results were not influenced by any individual study. Egger’s test (p=0.8984) and a funnel plot indicated no publication bias (Figure 3B).

**Figure 3:** (**A**) Forest plot for hypertension. (**B**) Funnel plot for hypertension.

### Diabetes and the severity of COVID-19

Thirty-two studies analyzed the association between diabetes and severe COVID-19. The pooled OR is shown in Figure 4A, which demonstrates that diabetes increased the risk of severe COVID-19 roughly 2.3-fold (random-effects model, OR=2.34, 95% CI: 1.79-3.05). The heterogeneity among the studies was high (I^2^=59%, p<0.01). A sensitivity analysis revealed that the results were not influenced by any individual study.

**Figure 4:** (**A**) Forest plot for diabetes. (**B**) Funnel plot for diabetes. (**C**) Funnel plot after used the trim-and-fill method for diabetes.

Publication bias was assessed using a funnel plot (Figure 4B) and Egger’s test, both of which revealed publication bias in this analysis (Egger’s test, p=0.0497). The trim-and-fill method was used to deal with the publication bias (Figure 4C). After the addition of seven studies, the combined-effect OR in the random-effects model was 1.7649 (95% CI: 1.32-2.36). The lack of obvious change indicated that the publication bias had little effect on the results, and the results were relatively stable.

## DISCUSSION

Cardiovascular diseases and diabetes are the most prevalent chronic diseases globally. During this ongoing pandemic, large numbers of people with these underlying conditions are inevitably going to contract COVID-19. The present systematic analysis summarized the results of 35 studies from December 2019 to July 5, 2020, and demonstrated that CHD, hypertension and diabetes each increased the risk of severe COVID-19 at least two-fold.

Regarding CHD, our meta-analysis of 25 qualifying studies indicated that the risk of developing severe COVID-19 was three times higher in patients with pre-existing CHD than in those without. Several possible explanations have been proposed for the impact of cardiovascular diseases on the progression of COVID-19 [40]. First, the acute pulmonary infection associated with COVID-19 may cause cardiac injury by inducing myocarditis [41], thus reducing systolic function and promoting heart failure. Second, the systemic inflammatory response to COVID-19 may cause coronary plaque rupture or erosion in patients with pre-existing CHD and thus induce acute coronary syndrome. Third, COVID-19-induced hypoxemia may trigger atrial fibrillation in elderly patients with cardiovascular diseases. The clinical presentation of COVID-19 may be similar to that of acute coronary syndrome or decompensated cardiovascular disease if it includes dyspnea and fatigue, and this may lead to misdiagnosis at the early stages of infection, thus delaying medical intervention.

The article "Impact of cardiovascular and metabolic diseases on the severity of COVID-19: a systematic review and meta-analysis" was published in 2020. Journal: Aging (Albany NY).

Our meta-analysis also demonstrated that the risk of developing severe COVID-19 was at least two times greater in patients with hypertension than in those without. It has been postulated that the progression of COVID-19 into severe COVID-19 in patients with hypertension may be due to prior and concomitant use of angiotensin converting enzyme (ACE) inhibitors or angiotensin II receptor blockers (ARBs) [42]. This proposed mechanism is based on the notion that ACE inhibitors and ARBs upregulate the expression or prevent the degradation of angiotensin II converting enzyme (ACE2), a receptor with high binding affinity for SARS-CoV-2. However, as of now, there is no reliable scientific basis or clinical evidence to support this view. Thus, it is necessary to further explore the potential impact of ACE inhibitors and ARBs on the pathogenesis and prognosis of COVID-19.

In this meta-analysis, we also found that the risk of severe COVID-19 was nearly two-fold higher in patients with diabetes than in those without. ACE2, the entry receptor for SARS-CoV-2, is expressed in various tissues, including the lungs, heart, renal tubules, small intestinal cavity surface and blood vessels [43]. Many drugs used by diabetic patients can increase the expression of ACE2, including glucagon-like peptide-1 agonists and statins [44]. The increased expression of ACE2 in multiple tissues of diabetic patients may increase the risk of COVID-19 infection. In addition, uncontrolled hyperglycemia can promote abnormal ACE2 glycosylation in the lungs, nasal airways, tongue and oropharynx, potentially increasing the binding sites of SARS-CoV-2 and the severity of the disease [45]. The mortality rate of COVID-19 was reported to be 7.6% in diabetic patients, but only 0.9% in patients without comorbidities [16]. Insulin resistance and uncontrolled blood glucose are important contributors to the deterioration of COVID-19. In severe COVID-19 patients, blood glucose levels were found to be increased to varying degrees in patients with diabetes [46]. Therefore, strict control of blood glucose may be critical for improving the clinical results of COVID-19 patients. However, it is worth noting that the mean age in our analysis was middle-aged, and it is highly likely that middle-aged patients with CHD, hypertension or diabetes have other diseases or bad habits. Thus, further study is needed to determine whether bad living habits aggravate COVID-19.

The article "Impact of cardiovascular and metabolic diseases on the severity of COVID-19: a systematic review and meta-analysis" was published in 2020. Journal: Aging (Albany NY).

Our heterogeneity analysis revealed moderate heterogeneity among the CHD studies and high heterogeneity among the hypertension and diabetes studies. Sensitivity analyses indicated that the results were not influenced by any individual study. When we excluded samples one by one to observe the dynamic changes in the meta-analysis, the results were not altered significantly, suggesting that the data were more stable after they were merged and that a random-effects model could be used. However, the results should be interpreted carefully due to their high heterogeneity.

There were several possible sources of heterogeneity in this study. 1. The quality of the available scientific literature for this meta-analysis was not ideal, as all the studies were large observational case series; however, due to the rapid spread of COVID-19, randomized controlled trials and prospective observational studies have not been conducted so far. 2. The results of this study demonstrated that patients with CHD, hypertension and diabetes were at increased risk for severe COVID-19 among hospitalized patients; however, 70-80% of COVID-19 patients may be asymptomatic or not require in-patient care. Further observational studies involving asymptomatic and mildly symptomatic patients not requiring hospitalization will be needed to determine the true magnitude of the effect of pre-existing CHD and metabolic diseases on COVID-19 severity. 3. Most of the patients were from Asia, although we included data from seven countries. As COVID-19 spreads globally, further study will be needed to determine whether there are ethnic differences in risk. 4. All the studies were clinical case observations, so there may have been heterogeneity in whether or for how long patients were followed up. 5. COVID-19 is an infectious disease that spread in a sudden worldwide outbreak. Thus, in sharing patient data for the first time, many researchers did not describe the diagnostic criteria for basic diseases such as CHD, hypertension and diabetes in detail, or did not fully consider the staging, severity, blood glucose control or blood pressure control of patients with these underlying diseases, leading to heterogeneity. Despite these limitations, this meta-analysis demonstrated that hospitalized patients with pre-existing CHD, hypertension and diabetes were at two- to three-fold higher risk for developing severe COVID-19 than those without these diseases.

The article "Impact of cardiovascular and metabolic diseases on the severity of COVID-19: a systematic review and meta-analysis" was published in 2020. Journal: Aging (Albany NY).

The results of this meta-analysis emphasize the importance of strictly limiting the spread of COVID-19 in patients with underlying cardiovascular and metabolic diseases, as they are the most vulnerable group. Clinicians should be aware of the approximately two- to three-fold higher risk of severe COVID-19 in these patients. Since elderly patients, smokers and patients with lung diseases are also more likely than others to progress to severe COVID-19 [47], clinicians should consider the patient’s age, underlying diseases, smoking status and other comprehensive factors when evaluating the prognosis of COVID-19. In addition, from a public health perspective, patients with co-morbid cardiovascular and metabolic conditions should be especially careful about hand hygiene and personal protection measures. Better control of blood glucose and blood pressure may improve the course of COVID-19, but further research is needed.

In summary, pre-existing cardiovascular and metabolic diseases increased the likelihood of severe COVID-19 and thus may promote a poor prognosis in COVID-19 patients.

## MATERIALS AND METHODS

### Data source, search strategy and inclusion criteria

We carried out a comprehensive, systematic literature search in five online databases (PubMed, Cochrane, Web of Science, WanFang Data and CNKI) from December 2019 to July 5, 2020 to identify potential studies. The search terms and relative variants used were as follows: "COVID-19" OR "2019 novel coronavirus infection" OR "coronavirus disease 2019" OR "2019 novel coronavirus disease" OR "coronavirus 2019" OR "2019-nCoV" OR "SARS-CoV-2" OR "COVID19" OR "coronavirus disease-19". The literature search included both English- and Chinese-language publications.

The titles, abstracts and full texts of all the documents identified through this search strategy were screened by two investigators (M.M. and QW.Z.). The reference lists of the review articles and research articles were also reviewed to detect other eligible documents. Studies were included if they reported diabetes, hypertension or CHD data in COVID-19 patients with or without a severe presentation. The definition of severe COVID-19 varied among the included studies. In this study, we defined COVID-19 as severe if the patient required intensive care, received mechanical ventilation or died, consistent with most of the articles. All the search results were evaluated according to the MINORS statement. Case reports, letters, non-human studies and studies without adequate information were excluded from the present meta-analysis.

The article "Impact of cardiovascular and metabolic diseases on the severity of COVID-19: a systematic review and meta-analysis" was published in 2020. Journal: Aging (Albany NY).

### Data extraction and quality assessment

The data extraction and literature quality evaluation were conducted independently by two investigators (M.M. and QW.Z.). Microsoft Excel was used to record all the available information, including baseline details, clinical data, the discharge rate and the fatality rate. Any disagreement was resolved by another investigator (B.W.).

### Data synthesis and statistical analysis

Microsoft Excel was used to analyze the combined results for patients with severe and non-severe disease. The meta-analysis was carried out using R software. Heterogeneity among the studies was assessed using the Cochran chi-square test and I^2^. When I^2^ was < 50%, a fixed-effects model was used, and when I^2^ was > 50%, a random-effects model was selected. If there was statistical heterogeneity in the results, a further sensitivity analysis was conducted to determine the source of the heterogeneity. After significant clinical heterogeneity was excluded, a random-effects model was used for meta-analysis. Funnel plots and Egger’s tests were used to detect publication bias. P<0.05 (two-sided) was considered statistically significant.
